# Prediction and Analysis of Length of Stay Based on Nonlinear Weighted XGBoost Algorithm in Hospital

This article has been retracted.

**DOI:** 10.1155/2021/4714898

**Published:** 2021-11-30

**Authors:** Yong Chen

**Affiliations:** The Affiliated Hospital of Chengde Medical College, Chengde, Hebei 067000, China

## Abstract

An improved nonlinear weighted extreme gradient boosting (XGBoost) technique is developed to forecast length of stay for patients with imbalance data. The algorithm first chooses an effective technique for fitting the duration of stay and determining the distribution law and then optimizes the negative log likelihood loss function using a heuristic nonlinear weighting method based on sample percentage. Theoretical and practical results reveal that, when compared to existing algorithms, the XGBoost method based on nonlinear weighting may achieve higher classification accuracy and better prediction performance, which is beneficial in treating more patients with fewer hospital beds.

## 1. Introduction

Hospital beds are one of the important medical resources, and these beds are usually used as an important indicator to measure the hospital service level, which can objectively reflect the development level of local medical system [1]. Due to the limited number of beds in most hospitals, the length of stay of patients is also closely related to the cost of hospitalization. Therefore, shortening the length of stay can not only increase the turnover of inpatients but also reduce the medical cost and the social medical burden [2]. For the medical system, it is very important to identify the relevant risk factors related to patient recovery and length of stay. Therefore, how to improve the allocation of hospital beds and alleviate the shortage of hospital beds is a major problem currently faced by hospital managers [3].

In the case of limited medical resources in hospitals and various uncertain factors in the treatment process, the problem of bed allocation has not been effectively resolved, and many hospital beds are still in short supply. Therefore, accurately predicting the length of stay will help to allocate hospital beds rationally and increase the utilization rate of beds [4].

The length of hospital stay is an important indicator of hospital management. Specifically, its prediction is to use statistical methods to summarize, analyze, and study its change rule and its distribution law and use machine learning algorithms [5, 6] to build models to predict the length of hospital stay [7]. Not only are these important key technology that need to be broken through in theoretical research, but they also have a certain engineering value for hospital bed scheduling arrangements and the improvement of hospital rescue capabilities [8]. Therefore, domestic and foreign scholars have conducted in-depth studies on the length of hospitalization of patients [9–11]. The research content is mainly divided into distribution fitting and parameter estimation. In the study of distribution fitting, some scholars use different distribution function to fit the length of stay of patients and compare their fitting effects. For example, Kong et al. [12] selected three widely used models, log-normal model, Weibull model, and Gamma model, used these three models to fit the distribution of length of stay in hospital, and evaluated the applicability of these three models. Coskun et al. [13] used the Markov process to analyze the hospitalization process of patient, which is divided into short, medium, and long hospital stays. The PH distribution is used to fit the distribution of the length of stay, and the maximum likelihood estimation method is used to obtain the estimated value of the parameter. The study also pointed out the inadequacy of choosing lognormal distribution and gamma distribution to fit the length of hospital stay. The empirical analysis results show that the use of the 6-phase Markov model to fit the length of stay is better than other distribution, but there is also overfitting phenomenon. Lazar et al. also described the hospitalization process as a Markov state so as to analyze the whole process of the patient from admission to discharge [14].

In the study of parameter estimation, most scholars adopt Expectation-Maximization (EM) algorithm to estimate the model parameters of the length of hospital stay. Reed et al. [15] used the convolution operation of two distributions to establish the model of hospitalization length variable, which is a well-known technology in the field of signal processing. The particularity of the model is that the variables of interest are considered to be the sum of two random variables with different distributions. One of the variables will take the recovery of patients from hospitalization as the model, while the other variable will take the hospital management process (such as discharge process) as the model. A novel improved model based on the classical maximum likelihood estimation and the EM algorithm is used to fit a group of real data in the hospital, where the results show that the effect of the proposed model is good. Since the average length of stay cannot well reflect the distribution characteristics, some references have studied the distribution of length of stay based on probability distribution. Ingeman et al. [16] studied the length of stay distribution of patients on the basis of the data of medical insurance center, fitted the probability distribution of length of stay with different probability distribution, and evaluated the fitting effect of different distributions according to KL indicators. Finally, the Coxian distribution is selected to divide the length of hospitalization into decision trees through three variables: age, gender, and hospital level. It provides an empirical basis for the traditional operations research model, verifies the common service time distribution of the queuing model through data, and provides help for hospital management decision-making.

Although these research methods based on inpatient data have achieved good results in the daily operation of the hospital, there is still an overfitting problem in establishing the superposition distribution based on a single continuous model. Therefore, some scholars began to design two or more distribution models to fit a group of hospitalization data, so as to make the fitting effect of the tail better. This overlay model not only makes the tail closer to the actual distribution but also better adjusts the fitting effect of other parts and solves the problem of insufficient fitting of a single distribution. Literature [16] established a prediction model of hospitalization duration based on SVM regression, analyzed the chaotic characteristics of time series from admission to discharge, and constructed the input vector of support vector regression model by phase-space reconstruction. Literature [17] adopts Naive Bayes (NB) methods to extract the characteristics of hospital resource data and patient data and establish the prediction model of length of stay. Literature [18] constructed the prediction model based on C4.5 decision tree. However, most of the existing research methods are for small data samples. When dealing with high-dimensional samples, data dimensionality reduction is required, which makes it easy to cause information loss and affect the accuracy of prediction [19].

The continuous emergence of big data analysis and processing methods in the field of data science provides an effective tool for massive data mining and data law learning. Extreme gradient boosting (XGBoost [20]) is a parallel integration algorithm suitable for large-scale datasets. It has the characteristics of multicore parallel operation, regularization promotion, and user-defined objective function, is suitable for processing structured data, and has high accuracy and interpretability. At present, XGBoost algorithm has been widely used in the field of data science [21–23].

In this paper, a nonlinear weight XGBoost algorithm is proposed to predict the length of hospitalization. Aiming at the problem of unbalanced data samples, the proposed algorithm uses the sample proportion and Sigmoid function to determine the sample weight and improve the objective function, so as to realize the effective learning of unbalanced data samples and improve the prediction accuracy.

The length of stay is an important basis for the rational allocation of hospital beds, and an important embodiment of the operation speed, medical level, and work quality of the hospital. However, the simple average length of stay cannot reflect its internal distribution characteristics, which is not reasonable as the basis of hospital bed management. In the case of asymmetric data distribution of patient length of stay, the decisions made by hospital managers based on the average length of stay may lead to unreasonable allocation of hospital beds and unnecessary losses. Therefore, this paper will select an appropriate model to fit the length of stay and find out the distribution law of the length of stay, which is of great significance to the improvement of hospital bed management and hospital rescue ability. In addition, by constructing the prediction model of inpatient length of stay, this paper discusses the application of the improved algorithm in the prediction of inpatient length of stay, hoping to bring some help to hospital managers in the scheduling and arrangement of hospital beds.

## 2. Related Works

XGBoost model is a machine learning algorithm implemented under the gradient boosting framework. It is a representative algorithm in boosting-based integrated algorithms [24]. The integrated algorithm constructs multiple weak-evaluators on dataset and summarizes the modeling results of all weak-evaluators to obtain better regression performance than a single model. The idea of XGBoost model is the process of continuously adding trees. Adding a tree every time is to learn a new function *f*(*x*) to fit the residual of the last prediction. After training, *k* trees will be obtained. Each tree will fall to a corresponding leaf node, and each leaf node corresponds to a score. Adding up the scores corresponding to each tree is the predicted value of the sample. In other words, XGBoost model generates a new tree through continuous iteration to fit the residual of the previous tree, as shown in Figure 1. With the increase of iteration times, the accuracy continues to improve. Therefore, XGBoost model can fit the inpatient data better, so as to reduce the prediction error and achieve high prediction accuracy.

The tree model used in this paper is CART regression tree model. It is assumed that there are *n* trees in the model, and the prediction results of the whole model on the sample can be shown in the following formula:

(1) $$\begin{array}{c} {\hat{y}}_{i}=\sum_{i=1}^{n}f_{i}\left(x_{i}\right),\;f_{i}\in F, \end{array}$$

where *n* is the number of trees, *f*_*i*_ is a function in function space *F*, ${\hat{y}}_{i}$ is the predicted value, *x*_*i*_ is the first *x*_*i*_ data entered by users, and *F* is all possible CART sets.

XGBoost has achieved good results in inventory and sales prediction, physical-event classification, web-text classification, customer-behavior prediction, click-through-rate (CTR) prediction, stock prediction, and other tasks, but it is rarely used in hospital length-of-stay prediction [25]. XGBoost provides scalable functions in all scenarios and can adopt external memory to ensure the calculation of big data, which can process a large amount of data with a small amount of node resources. XGBoost algorithm has the following advantages: XGBoost adds a regularization term to the objective function, reduces the variance of the model, makes the learned model simpler, and can effectively prevent overfitting; XGBoost carries out the second-order Taylor expansion of the loss function, which makes the model more accurate; XGBoost supports parallelization and column sampling, which has fast training speed [26]. Therefore, this paper will use XGBoost to predict the length of stay and treat more patients with limited medical beds.

Scholars at home and abroad mostly fit the distribution of inpatient length of stay [27]. However, the fitting of distribution only describes its distribution form through the length-of-stay data and cannot reflect what factors affect the length of stay of patients. This paper will use the improved XGBoost algorithm to establish the prediction model for the prediction of the length of stay. Firstly, preprocess the data, then extract the features from the patient data, take the medical features as the input variable to predict the length of stay, and finally realize the classified prediction of the length of hospitalization. In order to compare the prediction performance of different algorithms on the length of stay, the advantages and disadvantages of different methods in predicting the length of stay were experimentally discussed, so as to provide technical support for the prediction of the length of stay.

## 3. Nonlinear Weighted XGBoost Algorithm for Prediction of Length of Stay

As we all know, the traditional XGBoost algorithm aims to reduce the overall error, so it pays more attention to the classification and prediction performance of most class samples in the process of model learning, which will lead to the insufficient training of the classification performance of a few class samples [28, 29]. In the problem of length-of-stay prediction, this will also affect the prediction effect of the model for the allocation of hospital beds with relatively less frequency but more serious practical impact.

XGBoost model generates a new tree through continuous iteration to fit the residual of the previous tree. With the increase of iteration times, the accuracy continues to improve. At each iteration, the original model remains unchanged and a new function is added to the model. Since a function corresponds to a tree, the newly generated tree fits the residual of the last prediction. The iterative process is written as follows:

(2) $$\begin{array}{c} \left\{\begin{array}{c} {\hat{y}}_{i}^{\left(0\right)}=0,\\ {\hat{y}}_{i}^{\left(1\right)}=f_{1}\left(x_{i}\right)+{\hat{y}}_{i}^{\left(0\right)},\\ {\hat{y}}_{i}^{\left(t\right)}={\hat{y}}_{i}^{\left(t-1\right)}+f_{t}\left(x_{i}\right). \end{array}\right. \end{array}$$

The objective function of XGBoost is as follows:

(3) $$\begin{array}{c} F\left(y\right)=\sum_{i=1}^{n}l\left(y,\hat{y}\right)+\sum_{i=1}^{n}\Omega \left(f_{k}\right), \end{array}$$

(4) $$\begin{array}{c} \Omega \left(f_{k}\right)=\left.\gamma T+0.5\lambda \sum_{i=1}^{T}\varpi_{j}^{2}\right), \end{array}$$

where $l\left(y,\hat{y}\right)$ is used to measure the difference between the predicted score and the real score and ∑_*i*=1_^*n*^Ω(*f*_*k*_) is a regularization term. In (4), *T* is the number of leaf nodes, *r* is the score of leaf nodes, *γ* is used to control the number of leaf nodes, and *λ* is to ensure that the score of leaf nodes is not too large. The goal of regularization is to select a simple prediction function to prevent overfitting of the model [30]. When the regularization parameter is zero, XGBoost degenerates into a traditional boosting model. The iteration operation adopts the additive training to further optimize the objective function. In each iteration, the following strategy is adopted to update the objective function:

(5) $$\begin{array}{c} \tau^{\left(t\right)}=\sum_{i=1}^{n}l\left(y_{i},{\hat{y}}_{i}^{\left(t-1\right)}\right)+f_{t}\left(X_{i}\right)+\Omega \left(f_{t}\right). \end{array}$$

In order to minimize the objective function, XGBoost first expands the Taylor second-order expansion at *f*_*t*_=0 and extends the Taylor series of the loss function to the second-order. The objective function is approximate to the following equation:

(6) $$\begin{array}{c} \tau^{\left(t\right)}\approx \sum_{i=1}^{n}\left[l\left(y_{i},{\hat{y}}_{i}^{\left(t-1\right)}\right)+f_{t}\left(X_{i}\right)+0.5h_{i}f_{t}^{2}\left(x_{i}\right)\right]+\Omega \left(f_{t}\right). \end{array}$$

If the loss function values of each data are added up, the final objective function can be rewritten as follows:

(7) X≈obj∑i=1ngiftxi+0.5hift2xi+Ωft=λT+∑i=1ngft0.0.5Xi+0.5hift2xi+Ωft+0.5λ∑j=1Twj2=∑j=1T∑i∈Igiwj2+0.5∑i∈Ihi+λwj2+λT,

where *X*_obj_ is the loss function, $g_{i}=\partial {\hat{y}}^{t-1}l\left(y_{i},{\hat{y}}^{\left(t-1\right)}\right)$ is the first derivative, and $h_{i}=\partial^{2}{\hat{y}}^{t-1}l\left(y_{i},{\hat{y}}^{\left(t-1\right)}\right)$ is the second derivative.

It can be seen that (7) rewrites the objective function into a quadratic function about the leaf node fraction, and the optimal value is $g_{i}=\partial {\hat{y}}^{t-1}l\left(y_{i},{\hat{y}}^{\left(t-1\right)}\right)$, so objective function values can be obtain as follows:

(8) $$\begin{array}{c} w_{j}^{*}=-\frac{G_{j}}{\left(H_{j}+\lambda \right)},\\ X_{\text{obj}}=-0.5\sum_{j=1}^{T}\frac{G_{j}}{\left(H_{j}+\lambda \right)}+\lambda T, \end{array}$$

where *G*_*j*_=∑_*i*∈*I*_*g*_*i*_*H*_*j*_=∑_*i*∈*I*_*h*_*i*_.

It can be seen that the weight *w*_*j*_^*∗*^ will also affect the prediction effect of the model for the allocation of hospital beds with relatively less frequency but more serious practical impact. Therefore, this paper proposes a nonlinear weighting method to improve the performance of XGBoost model under data imbalance. The basic idea is to use heuristic function to nonlinear weight different categories of samples, and the number of samples is negatively correlated with the sample weight. The weight can be calculated as follows:

(1) Calculate the sample proportion.
  (9) $$\begin{array}{c} v_{k}=\frac{d_{k}}{D}, \end{array}$$
where *D* is the total number of samples, *d*_*k*_ is the number of samples of the *k* − th categories, and *v*_*k*_ is the proportion of the *k* − th categories sample in the total samples.
(2) Calculate the nonlinear weighting function.

Generally speaking, the weighting idea based on sample proportion can use the reciprocal of *v*_*k*_ in (10) as the weight. Although the reciprocal of *v*_*k*_ can improve the weight of a few samples, the weight of the categories accounting for the majority of samples decreases greatly, which may lead to excessive weight difference. In addition, if the proportion of most samples is much higher than that of a few samples, the weight of most samples may be very small, and the weight of a few samples may be too high, which may lead to low model training efficiency. Therefore, a nonlinear weighting function based on sample proportion is proposed in this paper.

(10) $$\begin{array}{c} w_{k}=0.5+\frac{\alpha }{\left(1+e^{v_{k}}\right)}. \end{array}$$

The nonlinear weighting function shown in (9) has two advantages: (1) the weighting function based on Sigmoid function is smooth and differentiable; (2) since too small weight will affect the training efficiency of the model and lead to overfitting, the constant 0.5 is added to the weighting function shown in (9) which can ensure that the weight will not be too small. According to (7), the value range of the function is [0.5+*α*/(1+*e*), 0.5+*α*/2], where *α* is the weight range control parameter.

Negative-log-likelihood (NLL) loss function is selected as the loss function to predict the length of stay. For samples *x* with the *k* − th categories, the NLL-based loss function can be denoted as $l\left(y_{i},{\hat{y}}_{i}\right)=-\sum_{k}y\left(k\right)\log\hat{y}\left(k\right)$. Therefore, the difference between the predicted score and the real score can be rewritten as follows:

(11) $$\begin{array}{c} l\left(y_{i},{\hat{y}}_{i}\right)=-w_{k}\log\hat{y}\left(k\right). \end{array}$$

In this paper, a hospital length-of-stay prediction algorithm based on nonlinear weighted XGBoost algorithm is proposed. The algorithm is divided into model training and test verification stages. In the model training stage, a new classifier is gradually added to fit the training error in the current iteration and optimize the fitting effect of the model on the training samples [15, 31]. In the test verification stage, the test set is used to verify the classification prediction performance of the model. The algorithm flow is shown in Table 1.

## 4. Experiment Results and Analysis

### 4.1. Parameter Settings

In our experimental, there are 114,209 real patient datasets from an open-source database, where 75% of them are training sets and 25% are test sets. In order to compare the model performance, the nonlinear weighted XGBoost algorithm is compared with Naive Bayes (NB) [32], decision tree (DT) [33], SVM [34], KNN [32], and XGBoost algorithm [20].

XGBoost algorithm has many parameters. Generally speaking, the initialization settings of parameters are as follows: *n_estimators, Gamma, Subsample, colsample-bytree*, and *learning rate* are set to 1000, 0, 0.8, 0.8, and 2, respectively. To improve the generalization ability of the model, optimizing the model parameters is also an essential step.

As for our improved XGBoost, three parameters need to be determined in the process of the length-of-stay prediction and have a great impact on the performance, including the learning rate, the maximum height of the tree, and the random sampling ratio. Since the maximum height of the tree affects the final result, this parameter should be tuned first. The tuning method first gives an initial value to other parameters, where important parameters are set to common typical values. Other parameters are set to default values.

In the model training stage, the grid search method is used to search all possible parameter combinations of each algorithm. For each parameter combination, the 3-fold cross validation experiment is used to determine the optimal parameters of each algorithm according to the cross validation results. The experimental algorithm is mainly implemented based on Python 3.7.7 and scikit-learn toolkit, and the hardware configuration is Intel Core i5-8300h CPU@2.3 GHz processor, 16-G memory. The parameters setting for different classifiers can be found in Table 2.

### 4.2. Data Preprocessing

As we all know, it is very important to select appropriate influencing factors in the prediction system for patient length of stay. Too few parameters will easily lead to overgeneralization, and the omission of key information will increase the error of final prediction. Too much parameters will increase the complexity of the model, and in the same case, the increase of the complexity of the model will often reduce the accuracy of the final result. Therefore, this paper tries to find a balance between the two in preprocessing stage so as to achieve satisfactory results: firstly, the selected influencing factors must not be too few and must be able to fully represent the problem. Secondly, the selected factors should not be too many; at least irrelevant influencing factors cannot be included. Similar to literature [23], we processed the adopted dataset.

### 4.3. Evaluation Indexes

In order to evaluate the performance of different models, this paper compares the performance of different models based on the relevant statistical indexes and performance curves of confusion matrix, including accuracy (ACC), Root Mean Square Error (RMSE), F1-score, and kappa coefficient. Performance curves include receiver operating characteristic (ROC) curve, precision recall (PR) curve, and learning curve.

ROC curve and PR curve can intuitively evaluate the performance of the classifier, where the ROC curve reflects the relationship between the true positive rate (TPR) and the false positive rate (FPR), and the PR curve reflects the relationship between the accuracy rate and the recall rate. At the same time, the classification performance of the model can be evaluated by comparing the size of the Area under the Curve (AUC) of different models. The true positive rate and false positive rate are shown as follows:

(12) $$\begin{array}{c} \text{FPR}=\frac{\text{FP}}{\text{FP}+\text{TN}}\times 100\%,\\ \text{TPR}=\frac{\text{TP}}{\text{TP}+\text{FN}}\times 100\%. \end{array}$$

### 4.4. Performance Analysis

#### 4.4.1. Distribution for Length of Stay

Our proposed nonlinear weighted XGBoost can rank the relative importance of feature variables. It reflects the value of each feature variable when training the model. The greater the value of the feature variable when training the model, the higher its relative importance. The results showed that the variables that had the greatest impact on the length of stay were the number of operations, transfer status, and age. From a common sense point of view, the more surgeries there are, the longer it takes to be hospitalized for treatment. The older the age, the longer the hospital stay, which is also consistent with the results of medical research. In addition, the status of transfer, discharge outcome, and discharge diagnosis are closely related to the length of stay in the hospital. However, factors such as gender and number of rescues do not have much influence on the length of the patient's hospital stay. The analysis of important characteristics not only is of great significance for predicting the length of stay but also can bring important reference opinions to medical staff.

A descriptive statistical analysis was made on the length of stay from the perspective of the gender of the patients. The results of the statistical analysis are shown in Table 3.

As shown in Table 3, the shortest and longest hospitalization days of patients in the hospitalization data record are 1 day and 73 days, where 99.49% of the patients were hospitalized for less than 25 days. The average length of stay was 9.1 days, and the median length of stay was 8 days. The total length of hospitalization skewness coefficient was 2.289 and kurtosis coefficient was 9.55. Therefore, the length of stay distribution of patients showed a right deviation.  Figure 2 shows the distribution of the length of stay of patients, where there is a “long tail” phenomenon in the number of samples with different length of stay. In other words, the distribution of sample is unbalanced. Due to the difference in the number of samples, the “normal” category with a large number will be fully trained, while the number of samples with long length is relatively small.

From the perspective of gender, there are 1028 male patients, accounting for 57.1% of the total number, and 958 female patients, accounting for 42.9% of the total number. The ratio of male to female patients is 1.3 : 1. The youngest male patient was 11 years old, the oldest was 91 years old, and the average age was 62 years old. The youngest female patient was 7 years old, the oldest was 89 years old, and the average age was 65 years old. Overall, the average length of stay of male patients was 0.93 days longer than that of female patients and was greater than the overall average length of stay. The skewness coefficients of male and female patients were positive, so the length of hospitalization showed a right skewness. The kurtosis of the length of stay of female patients is much greater than that of male patients, and greater than the overall kurtosis.

#### 4.4.2. Predictive Performance Analysis

After feature processing, the characteristic variables of patient hospitalization are used as the feature input of machine learning model, and the model is trained, verified, and predicted on the training set and test set. In order to verify the effect of the improved CGBoost algorithm on predicting the length of stay, we compare it with the traditional classical algorithm and analyze the performance indicators of the prediction models for different algorithms.

Table 4 shows the quantitative prediction indicators of different algorithms. It can be seen that the accuracy (ACC), Root Mean Square Error (RMSE), F1-score, and kappa coefficient of our proposed algorithm are 0.8211, 1.823, 0.8501, and 0.8122, respectively, which has good practical performance. In other words, it is indicated that our proposed XGBoost model is feasible in predicting the length of stay. The accuracy (ACC), Root Mean Square Error (RMSE), F1-score, and kappa coefficient of the decision tree algorithm are 0.824, 0.806, 0.829, and 0.818, respectively. The prediction effect is general. The performance of decision tree model in predicting the length of stay is not as good as our improved XGBoost model. The quantitative performance indexes of the KNN are 0.811, 1.721, 0.773, and 0.848, respectively. The prediction accuracy is not as high as XGBoost model and decision tree model. However, the AUC of the model is higher, which shows that the logical regression model is more robust than the decision tree model. The AUC value and accuracy of the XGBoost algorithm are higher than those of decision tree and KNN, which means that the prediction effect of XGBoost model is better and the stability of the model is stronger.

According to the above results, the hospital length-of-stay prediction of our proposed model has achieved good results. Compared with the traditional model, it has a good improvement in stability and accuracy and has a certain practical value.

Figure 3 shows the comparison of AUC values of classifier PR curve and PR curve. It can be seen that our proposed XGBoost algorithm has higher AUC values and is better than other comparative classifiers.

As can be seen from Figure 4, our proposed algorithm has the fastest convergence accuracy, followed by *XGBoost algorithm* and *Naive Bayes* algorithm, respectively. *KNN* algorithm has the lowest score on the training set and cross validation set, and the other algorithms have the overfitting state for unbalance data. At the same time, it can be seen from Figure 4 that our algorithm has the highest score on the cross validation set, which is consistent with the experimental results in Table 4.

According to the results of various indicators and performance curves, it can be seen that our proposed algorithm can achieve good classification and prediction performance for length of stay in hospital. The nonlinear weighting method can not only ensure the overall accuracy but also improve the classification accuracy. In addition, the improved XGBoost algorithm also shows its advantages in convergence speed and learning ability compared with traditional classifiers in Figure 5. It should be noted that the proposed algorithm increases the weight control parameter *α* compared with XGBoost algorithm, and there are five possible values in its parameter range. Therefore, in the process of parameter optimization, the parameter combination of our algorithm is five times that of XGBoost algorithm, which requires more parameter optimization time.

In general, the purpose of this paper is to use the proposed algorithm to predict the length of hospitalization based on the limited bed resources of the hospital. We need to not only obtain accurate prediction accuracy but also obtain the optimal bed scheduling.

## 5. Conclusion

The resources that hospitals can provide are often unable to meet the needs of hospitalization. Accurately predicting the number of days a patient will stay in the hospital can improve the efficiency of hospital operations. This paper proposes to use a nonlinear weighted XGBoost algorithm to predict and analyze patient hospitalization data. Due to the imbalance of real case data, the XGBoost algorithm used improves the objective function based on the idea of sample ratio and nonlinear weighting, which improves the classification and prediction ability of the algorithm in the case of imbalanced data samples. In order to verify whether the prediction performance of the proposed algorithm can meet actual application requirements, the experimental part uses multiple comparison algorithms for experimental verification. The experimental results show that the algorithm proposed in this paper has obvious advantages for unbalanced data. This further shows that the research work in this paper can be applied to real application. There are still some shortcomings in this research. For large datasets, the processing performance of the algorithm used is not good. However, with the passage of time and the increase in case data, the amount of data will inevitably increase gradually. How to improve the processing time and accuracy of the algorithms used for big data is the direction that our team will continue to study in the future. In addition, we also need to consider how to use predictive information to optimize the use of resources in hospitals when encountering some emergencies and the surge in case data. This is what we need to study in the future.

## Figures and Tables

**Figure 1:** Framework of XGBoost model.

**Figure 2:** Distribution of the length of stay of patients.

**Figure 3:** Comparison of ROC curve for different models.

**Figure 4:** Comparison of PR curve for different models.

**Figure 5:** Comparison of learning curve for different models.

**Table 1:** Pseudocode for nonlinear weighted XGBoost algorithm.

Model: nonlinear weighted XGBoost algorithm
Input: high-dimensional patient medical data
Output: hospital length-of-stay
*X*_Obj_ ← 0, *G* ← ∑_*i*∈*I*_*g*_*i*_, *H* ← ∑_*i*∈*I*_*h*_*i*_, and ${\hat{y}}_{i}^{\left(0\right)}=0$
For *k* = 1 to *m* do
*G*_*L*_ ← 0, *H*_*L*_ ← 0
For *j* in sorted(*I*, by *x*_*kj*_)
${\hat{y}}_{i}^{\left(t\right)}\leftarrow {\hat{y}}_{i}^{\left(t-1\right)}+f_{t}\left(x_{i}\right)$
Ω(*f*_*k*_) ← *γT*+0.5*λ*∑_*i*=1_^*T*^*ϖ*_*j*_^2^)
*w*_*k*_ ← 0.5+*α*/(1+*e*^*v*_*k*_^)
$l\left(y_{i},{\hat{y}}_{i}\right)\leftarrow -w_{k}\log\hat{y}\left(k\right)$ *X*_obj_←∑_*j*=1_^*T*^[∑_*i*∈*I*_*g*_*i*_*w*_*j*_^2^+0.5(∑_*i*∈*I*_*h*_*i*_+*λ*)*w*_*j*_^2^]+*λT*
End
End

**Table 2:** Parameters setting for different classifiers.

The adopted classifiers	The setting of the predefined parameters
The proposed method	Number of trees: [10, 30, 50, 100]
	Maximum depth of tree: [3, 5, 8, 10]
	Minimum leaf node weight sum: [1, 3, 6, 9]
	Learning rate parameters: [0.05, 0.1, 0.15, 0.2]

Naive Bayes	Weight control parameters: [0.5, 1, 1.5, 2, 2.5]

XGBoost	Default parameters
	Smoothing parameters

SVM	Kernel function: RBF
	Penalty coefficient: [0.01, 0.1, 1, 10]
	Kernel parameter: [0.01, 0.001, 0.0001]

KNN	Number of nearest neighbors: [3, 5, 8, 10]
	Maximum number of leaves: [5, 8, 10, 30]

Decision tree	Number of trees: [10, 30, 50, 100]
	Maximum depth range: [3, 5, 8, 10]
	Learning rate range: [0.05, 0.1, 0.15, 0.2]

**Table 3:** Gender distribution.

	Number of patients	Mean	Median	Standard deviation	Kurtosis	Skewness
Total	1986	9.10	8	14.25	9.55	2.289
Male	1028	9.69	8	14.68	7.18	2.158
Female	958	8.26	9	13.01	15.67	2.731

**Table 4:** Quantitative prediction indicators of different algorithms.

Model	ACC	RMSE	F1-score	Kappa coefficient
Naive Bayes	0.7912	2.211	0.725	0.8017
Decision tree	0.8247	1.885	0.829	0.8182
SVM	0.8661	1.592	0.865	0.8611
KNN	0.8117	1.721	0.773	0.8482
XGBoost	0.7958	1.807	0.782	0.8251
The proposed model	0.8211	1.523	0.851	0.8622

## Data Availability

The dataset used to support the findings of this study are available from the corresponding author upon request.
